The article "Ethyl Acetate Fraction from Hedyotis diffusa plus Scutellaria barbata Suppresses Migration of Bone-Metastatic Breast Cancer Cells via OPN-FAK/ERK/NF-κB Axis" was published in 2020. Journal: Evid Based Complement Alternat Med.

# Ethyl Acetate Fraction from *Hedyotis diffusa* plus *Scutellaria barbata* Suppresses Migration of Bone-Metastatic Breast Cancer Cells via OPN-FAK/ERK/NF-*κ*B Axis

**DOI:** 10.1155/2020/3573240

**Published:** 2020-04-10

**Authors:** Ting Fang, Ying-Xuan Yan, Yue Yang, Ya-Xin Lv, Qing-Qi Chang, Dan-Dan Zhang

**Affiliations:** ^1^Institute of Interdisciplinary Integrative Medicine Research, Shanghai University of Traditional Chinese Medicine, Shanghai 201203, China; ^2^School of Pharmacy, Fujian University of Traditional Chinese Medicine, Fujian 350122, China; ^3^School of Pharmacy, Shanghai University of Traditional Chinese Medicine, Shanghai 201203, China

## Abstract

*Hedyotis diffusa* plus *Scutellaria barbata* is a couplet of medicinal that has been commonly used to treat inflammation-related diseases and various types of tumors. However, the effect of this couplet on tumor cell migration has not been elucidated. With the aid of MCF-7-BOM, a bone-metastatic subline of ER + breast cancer MCF-7, we showed that ethyl acetate fraction extracted at an equal weight ratio of *Hedyotis diffusa* plus *Scutellaria barbata* (EA11) inhibited cell migration of MCF-7-BOM in a concentration-dependent manner. To define the underlying molecular mechanism, we revealed that EA11 reduced the expression of osteopontin (OPN) and interfered with the FAK/ERK/NF-*κ*B signaling pathways, which are both critical for breast cancer bone metastasis. This study strongly suggested EA11 may represent a potential therapeutic agent against bone metastasis of breast cancer.

## 1. Introduction

Metastasis is a severe threat to the survival of breast cancer patients worldwide [1, 2], and bone metastasis occurs in approximately 65% of advanced breast cancer patients. Patients with bone metastasis suffer from bone pain, pathological fractures, hypercalcemia, and spinal cord compression, and the five-year survival rate is about 20% [3, 4]. Conventional therapeutic approaches against bone metastasis include radiotherapy, chemotherapy, targeted therapy, endocrine therapy, and bone-modulating drug therapy. However, the effectiveness of the currently available interventions is limited [5].

Osteopontin (OPN), which is a secreted glycol-phosphoprotein and encoded by gene SPP1, participates in bone matrix mineralization and reabsorption process in bone remodeling. Abnormal expression of OPN is detected in a variety of tumors (breast cancer, prostate cancer, lung cancer, gastric cancer, and melanoma) and is closely associated with the initiation, metastasis, and prognosis of breast cancer [6, 7]. Experimental evidence also supports the role of OPN in bone metastasis of breast cancer. In a recent study, the activation of the focal adhesion kinase (FAK) pathway was reported as an inevitable event of OPN-induced cell migration [8]. OPN has also been found to activate ERK1/2 through its binding to *α*v*β*3 integrin [9], which in turn promotes breast cancer progression. Moreover, OPN has been shown to augment cancer cell invasiveness via the NF-*κ*B-mediated signaling mechanism [10]. These findings suggest that targeting OPN-associated signaling pathways may be a potential therapeutic strategy against bone metastasis of breast cancer [11, 12].

Traditional Chinese medicine (TCM) has been widely used as an essential adjuvant treatment for malignant tumors in China. *Hedyotis diffusa*, a plant of the Rubiaceae family, contains flavonoids, polysaccharides, triterpenoids, sterols, and terpenoids. Many ingredients of *Hedyotis diffusa* possess antioxidation, anti-inflammatory, and antitumor activities. *Hedyotis diffusa* is commonly used in the treatment of breast cancer, colon cancer, liver cancer, and lung cancer [13–15]. *Scutellaria barbata* belongs to the Labiatae family and also displays antitumor activity. Similarly, *Scutellaria barbata* is also commonly used to treat various tumors [16, 17]. Especially, *Hedyotis diffusa* plus *Scutellaria barbata* are often used as a couplet medicine to treat various inflammation-related diseases and cancers [18, 19].

We previously reported that EA11 possesses potent anti-inflammatory activity [20]. As chronic inflammation is one of the hallmarks of cancer, we investigated the effects of EA11 on the migration of MCF-7-BOM cells and further explored the pertinent molecular mechanism.

## 2. Materials and Methods

### 2.1. Reagents and Chemicals

*Hedyotis diffusa* and *Scutellaria barbata* were purchased from Shanghai Yanghetang Pharmaceutical Company (Zhangjiang High-Tech Park, Shanghai, China) and confirmed by Shanghai Institute for Food and Drug Control (SIFDC). MCF-7-BOM was provided by Dr. Yu-dong Zhou (University of Mississippi, USA). Dulbecco's modified Eagle's medium (DMEM) medium-dry powder, fetal bovine serum, and 0.25% trypsin were obtained from Gibco BRL (Grand Island, NY, USA). 3-(4,5-Dimethylthiazol-2-yl)-2,5-diphenyltetrazolium bromide (MTT) and dimethyl sulfoxide (DMSO) were purchased from Sigma-Aldrich (St. Louis, MO, USA). The sources of used antibodies are the anti-OPN antibody (22952-1-AP) from Proteintech (Chicago, IL, USA), anti-p-FAK (BS4718) from Bioworld Technology (St. Paul, MN, USA), and anti-FAK (#3285), anti-NF-*κ*B (#3033), anti-p-NF-*κ*B (#8242), anti-ERK1/2 (#9102), and anti-p- ERK1/2 (#9101) from Cell Signaling Technology (Boston, MA, USA).

### 2.2. Preparation and Identification of the Main Components of EA11

EA11 was prepared as we previously described and further characterized by HPLC [20].

### 2.3. Cell Culture

MCF-7-BOM cells were cultured in DMEM medium containing 10% fetal bovine serum and incubated in a 37°C, 5% CO_2_ incubator (Thermo, Waltham, MA, USA). Cells were subcultured once every 2-3 days.

### 2.4. Cell Viability Assay

MCF-7-BOM cells were seeded in a 96-well plate at a density of 2 × 10^3^ cells per well overnight. Cells were then treated with EA11 (0, 12.5, 25, 50, 100, and 200 *μ*g/ml) or 0.25% DMSO (vehicle control) for 72 h followed by adding 20 *μ*l of 5 mg/ml MTT solution into each well. After 4 h incubation, culture supernatants in wells were removed, and 100 *μ*l of DMSO solution was added to dissolve the crystals completely. The optical density values at 490 nm were measured by a plate reader (Molecular Devices, CA, USA).

### 2.5. Wound-Healing Assay

MCF-7-BOM cells were seeded in a 6-well plate at a density of 6 × 10^5^ cells per well overnight. A scratch was generated with a sterile pipet tip followed by several washes to remove dislodged cells. Cells were then cultured in the complete medium containing 0, 25, and 50 *μ*g/ml of EA11 and photographed at 0, 24, and 48 h under an optical microscope (100x) (Olympus, Tokyo, Japan). Cell migration was determined by monitoring the sizes of gaps.

### 2.6. Transwell Migration Assay

MCF-7-BOM cells treated with or without EA11 treatment for 24 h were plated into the upper chamber (8 *μ*m pore size; Corning Incorporated, ME, USA) at 5 × 10^4^ cells per well, while 600 *μ*l serum-free medium was added into the lower chamber. After 24 h cell migration, cells in upper chambers were removed with cotton swabs, and cells on the lower surface of the chamber were fixed with 0.5% crystal violet. The photographs were taken under an optical microscope (200x), and cell migration was quantitated by counting stained cells.

### 2.7. Invasion Assay

To evaluate the invasiveness of MCF-7-BOM cells, cells were first treated with or without EA11 for 24 h and then added into the upper chamber of a Matrigel-coated Transwell plate (8 *μ*m pore size; Corning Incorporated, ME, USA) at the density of 2 × 10^5^ cells per well, while 600 *μ*l medium with 5% FBS was added to the lower chamber. After the 22 h invasion period, cells remaining in the upper chamber were removed with cotton swabs, while cells on the undersurface of upper chambers were stained with 0.5% crystal violet. The in vitro invasion is measured by counting stained cells under an optical microscope (200x).

### 2.8. Western Blotting Analysis

Cells were washed and lysed on ice using a protease-containing cell lysate (Beyotime Technology, Jiangsu, China). The protein concentration of each sample was determined by the BCA protein assay kit (Thermo Fisher Scientific, Waltham, MA, USA). Protein samples (30 *μ*g/lane) were separated on a 10% SDS-PAGE and transferred to the PVDF membrane. After blocking with 5% nonfat milk, membranes were blotted with the respective antibodies and visualized using ECL Western Blotting Detection Reagent (Millipore, Bedford, MA, USA) on the Tanon imaging system (Tanon, Shanghai, China).

### 2.9. Statistical Analysis

Statistical analyses were performed by ANOVA using SPSS version 20.0, and all experiments were repeated for at least three independent experiments. Results were presented as mean ± SD. The value of *P* < 0.05 was considered to be significant.

## 3. Results

### 3.1. Effect of EA11 on MCF-7-BOM Cell Growth

To determine the effect of EA11 on MCF-7-BOM cell growth, cells were treated with varying concentrations of EA11 for 72 h followed by MTT assay to measure cell growth. By comparing with the untreated cells, we observed that EA11 at 100 *μ*g/ml significantly inhibited the growth of MCF-7-BOM cells (*P* < 0.05) (Figure 1), indicating that EA11 at concentration <100 *µ*g/ml is little cytotoxic.

### 3.2. EA11 Inhibits MCF-7-BOM Cell Migration and Invasion In Vitro

As EA11 at concentration <100 *µ*g/ml is little cytotoxic, we investigated the effect of EA11 on cell migration at concentrations of 25 and 50 *μ*g/ml. Both wound-healing and Transwell assays showed that EA11 deterred migration of MCF-7-BOM cells in a dose- and time-dependent manner (*P* < 0.05) (Figure 2). In a parallel experiment, we examined the effect of EA11 on the invasiveness of MCF-7-BOM cells using Matrigel invasion chambers. While MCF-7-BOM cells readily invaded Matrigel, EA11 blocked the in vitro invasion of these cells in a concentration-dependent manner (*P* < 0.05) (Figure 3).

### 3.3. EA11 Downregulates the Expression of OPN in MCF-7-BOM Cells

OPN has been reported to be involved in the proliferation, migration, and invasion of breast tumor cells and associated with bone tumor microenvironment [21]. To determine whether EA11-led suppression in cell migration and invasion are functionally linked to OPN, we analyzed the effect of EA11 on OPN expression in MCF-7-BOM cells. Similarly, to what we observed with cell migration/invasion, western blot showed that EA11 dose dependently reduced the abundance of OPN in MCF-7-BOM (*P* < 0.05) (Figure 4).

### 3.4. EA11 Interferes with FAK/ERK/NF-*κ*B Signaling Pathways in MCF-7-BOM Cells

Binding of OPN to integrins has been shown to regulate migration and invasion of breast cancer cells, and activation of the focal adhesion kinase (FAK) signaling pathway is critical for OPN regulation of cell migration/invasion [8]. ERK/MAPK signaling pathway functions downstream of FAK to facilitate cell migration, while the enhanced level of OPN was reported to be correlated with elevated NF-*κ*B activity in breast and liver tumors [10]. To investigate the potential link between EA-induced reduction in OPN expression and these signaling pathways, we treated MCF-7-BOM cells with EA11 at concentrations of 0, 25, and 50 *μ*g/ml followed by western blotting to detect phosphor-FAK, phosphor-ERK, and phosphor–NF–*κ*B. Phosphorylation of FAK, ERK, and NF-*κ*B was readily seen in MCF-7-BOM cells. In contrast, EA11 diminished the phosphorylation levels of FAK, ERK, and NF-*κ*B (*P* < 0.05) (Figure 5), suggesting that interference of FAK/ERK/NF-*κ*B signalings by EA11 is most likely responsible for EA11-led suppression in OPN expression and cell migration/invasion.

## 4. Discussion

Late-stage of breast cancer often accompanies with clinical metastasis to the lung, liver, brain, and bone [22]. During bone metastasis, breast cancer cells have to undergo an invasion-transfer cascade to convert themselves to metastatic cells [23, 24]. Cancer cells often concentrate on the endosteal after reaching the bone site and then break the delicate balance between osteoblasts and osteoclasts in the bone microenvironment. The distortion of such a balance disrupts normal bone remodeling and integrity and finally leads to bone destruction [25, 26]. In the molecular level, abnormal osteoprotegerin (OPG)-RANKL ratio triggers a vicious circle of osteolytic metastasis [27, 28].

The level of OPN expression increases in breast cancer and prostate cancer patients with poor prognosis and shortened survival. Downregulating OPN expression has been shown to deter the progression and metastasis of breast cancer, indicating that OPN acts as a significant mediator of tumor progression and metastasis. The fact that OPN displays a particular affinity to the bone further highlights its importance in bone metastasis [7, 29, 30]. In this study, we showed that EA11 significantly decreased OPN expression in MCF-7-BOM cells and greatly inhibited cell migration and in vitro invasion.

NF-*κ*B activation is critical for various integrin signaling and tumor metastasis [10]. NF-*κ*B inhibitors have been shown to inhibit OPN-induced cell migration [9]. One of the examples is that treatment of A549 cells with NF-*κ*B inhibitor (PDTC) or IkappaB protease inhibitor (TPCK) blocked OPN-induced migration of lung cancer cells [31]. Recent studies have also shown that OPN can increase the levels of phosphor-FAK, AKT, and ERK in A549 cells, indicating that they might be mediators of OPN-led cell migration. Since OPN-stimulated phosphorylation of ERK is diminished by the FAK mutant, while FAK and ERK2 mutants can reduce OPN-induced NF-*κ*B activation, results from these studies suggest that a signaling axis consisting of FAK, ERK, and NF-*κ*B regulates OPN regulation of cell migration and invasion [9]. Our observation that EA11 inhibits breast cancer cell migration/invasion and interferes with the activation of the FAK/ERK/NF-*κ*B signaling pathway indicates that EA11 may be an active agent against bone metastasis of breast cancer cells.

## 5. Conclusions

Our results demonstrate that EA11 inhibited the migration of MCF-7-BOM cells. EA11-led inhibition in cell migration is most likely associated with the suppression of OPN expression and inactivation of FAK/ERK/NF-*κ*B signaling pathways. This study suggests that EA11 may represent as a potential therapeutic agent for the treatment of breast cancer bone metastasis.

## Figures and Tables

**Figure 1:** Effect of EA11 on the proliferation of MCF-7-BOM. MCF-7-BOM cells were seeded in a 96-well plate overnight. These cells were treated with EA11 (0, 12.5, 25, 50, 100, and 200 *μ*g/ml) or vehicle control for 72 h, and MTT assay was carried out. ^*∗∗*^*P* < 0.01 vs. vehicle.

**Figure 2:** Effect of EA11 on wound healing of MCF-7-BOM cells. (a) A scratch was generated with a pipette tip, and cells were grown with or without EA11 treatment at concentrations of vehicle, 25, and 50 *μ*g/ml. Images were taken at 0, 24 h, and 48 h under a phase-contrast microscope. (b) Cells were grown by treatment of EA11 at concentrations of vehicle, 25, and 50 *μ*g/ml. The mobility in 3 random fields of vehicle, 24, and 48 H treated with vehicle, 25, and 50 *μ*g/ml EA11. Data are means ± SD. *n* = 3. ^*∗*^*P* < 0.05, ^*∗∗*^*P* < 0.01 vs. vehicle.

**Figure 3:** Effect of EA11 on the migration and invasion ability of MCF-7-BOM cells. (a) Cells were treated with vehicle, 25, and 50 *μ*g/ml for 24 h followed by the analysis of cell migration using Transwell under a light microscope at 200x. (b) The migrated cells were counted at each group. (c) Cells were treated with vehicle, 25, and 50 *μ*g/ml for 22 h followed by the analysis of cell invasion using Matrigel-coated Transwell under a light microscope at 200x. (d) The invaded cells were counted at each group. ^*∗∗*^*P* < 0.01 vs. vehicle.

**Figure 4:** Effect of EA11 on the expression of the OPN protein. Following treatment of MCF-7-BOM cells with the vehicle, 25, and 50 *μ*g/ml of EA11, OPN protein was assessed by western blot. ^*∗∗*^*P* < 0.01 vs. vehicle.

**Figure 5:** Effect of EA11 on phosphorylation of FAK/ERK/NF-*κ*B signaling pathways. p-ERK, ERK, p-FAK, FAK, p-NF-*κ*B, and NF-*κ*B protein expressions were assessed by western blot following treatment of vehicle, 25, and 50 *μ*g/ml of EA11. ^*∗*^*P* < 0.05, ^*∗∗*^*P* < 0.01 vs. vehicle.

## Data Availability

The original data used to support the findings of this study are available from the corresponding author upon request.
